# Application Effect of Acupoint Massage on Zusanli on Premature Infants with Feeding Intolerance and Their Clinical Symptoms

**DOI:** 10.1155/2021/7772543

**Published:** 2021-12-09

**Authors:** Yueqiu Gong, Li Zhu

**Affiliations:** Department of Pediatrics, Suzhou Hospital of Traditional Chinese and Western Medicine, Suzhou 215101, Jiangsu Province, China

## Abstract

FI is mainly caused by functional disturbance in premature infants, which greatly poses a threat to their growth and development, so a large number of studies on the clinical features of FI should be conducted to provide theoretical support for treatment. The purpose of the study was to investigate the therapeutic effect of acupoint massage on Zusanli on premature infants with feeding intolerance (FI) and their clinical symptoms. A total of 60 premature infants with FI admitted to our hospital over the past two years were selected as the FI group, and another 60 premature infants without FI were selected as the control group. The birthweight and gestational age of the premature infants in the FI group were significantly lower than those in the control group (*P* < 0.001), whereas there were no significant differences in general information of the premature infants between the two groups (*P* > 0.05). Vomiting, abdominal distension, and gastric retention are the main clinical symptoms of premature infants with FI, and acupoint massage on Zusanli combined with routine treatment can effectively improve digestive function, relieve clinical symptoms, and shorten treatment time of premature infants with FI, which is worthy of application and promotion in clinical practice.

## 1. Introduction

Nowadays, the increasing number of newborn premature infants is varying from 10 to 20 million per year across the world, accounting for more than 10% of the overall live birth rate. Although advanced medical technologies have greatly saved more and more premature infants, their life quality is still not satisfactory, owing to the incomplete organ development, thus adversely affecting the growth and development of premature infants [1–3]. FI, as one of the most common conditions in premature infants, is mostly caused by poor development of digestive organs, and affected infants usually present with vomiting, abdominal distension, and gastric retention. Besides, in some cases, mental retardation also affects premature infants, further increasing the probability of death. Therefore, the academic community should pay more attention to further exploring the clinical symptoms of premature infants with FI to provide solid theoretical support for the selection of suitable treatment and drugs [4–7]. At present, erythromycin is the main drug for the treatment of FI in clinical practice, whose mechanism is to enhance gastrointestinal motility and subsequently relieve the symptoms of FI in affected infants; however, this drug can also increase the incidence of abdominal pain and abdominal distension, so combination therapy should be implemented to improve treatment effect of FI. Acupoint massage on Zusanli is an auxiliary intervention relying on the theory of traditional Chinese medicine, which serves the function of regulating spleen and stomach, and it is often used in the treatment of gastrointestinal diseases.

However, there are just few studies on the application of acupoint massage on Zusanli for the premature infants with FI; based on this, in this study, in order to investigate the therapeutic effect of acupoint massage on Zusanli on premature infants with FI and their clinical symptoms, 120 premature infants admitted to our hospital over the past two years were selected as the study subjects, and now the study results are reported as follows.

## 2. Materials and Methods

### 2.1. General Information

A total of 60 premature infants with FI admitted to our hospital over the past two years were selected as the FI group, and another 60 premature infants without FI were selected as the control group. At the same time, the FI group was divided into group A and group B, and there were no significant differences in the general information of the premature infants in the two groups (*P* > 0.05), which can be used as the study samples, as shown in Table 1. After that, the general information of the premature infants in both groups was compared and the clinical symptoms of the premature infants in the FI group were recorded and analyzed. Meanwhile, the FI group was randomly divided into group A and group B, in which the premature infants in group B were treated with erythromycin, while the premature infants in group A were treated with erythromycin combined with acupoint massage on Zusanli; then, the digestive function, observation indexes of intolerance, and other treatment indexes were all compared between group A and group B.

### 2.2. Inclusion Criteria

① Family members of the premature infants were informed of the purpose and process of the study and signed the informed consent. ② This study was approved by the Hospital Ethics Committee. ③ Premature infants had the gestational age of less than 37 weeks. ④ Premature infants had no infection. ⑤ Premature infants met the diagnostic criteria for FI.

### 2.3. Exclusion Criteria

① Premature infants had other organic diseases such as congenital gastrointestinal tract anomalies. ② Premature infants had inherited metabolic disorders.

### 2.4. Methods

#### 2.4.1. Information Collection

The general information of premature infants in the FI group and the control group was collected, and the clinical symptoms of the premature infants in the FI group were recorded and analyzed.

#### 2.4.2. Treatment Methods

The premature infants in group B received the nasal feeding of erythromycin (Sinopharm Group Sanyi Pharmaceutical Co., Ltd.; State Food and Drug Administration approval number: H34020307) every 6 hours, at 5 ml kg^−1^ d^−1^ [8–11], while based on the treatment in group B, the premature patients in group A were treated with acupoint massage on Zusanli by vertically kneading Zusanli acupoint with finger pulp for 5 min, twice a day [12–15].

### 2.5. Evaluation Indexes

① The general information of the premature infants such as gender, gestational age, weight, maternal age, delivery mode, and complications during pregnancy was compared between the FI group and the control group. ② Clinical symptoms of the premature infants in the FI group. The gestational age of the premature infants was divided into three levels (<30 weeks, 30–35 weeks, and 36–37 weeks), the weight of the premature infants was divided into three levels (<1500 g, 1500–2500 g, and >2500 g), and the breastfeeding initiation time of the premature infants was divided into two levels (<72 h and ≥72 h). We also compared the clinical features such as vomiting, abdominal distension, gastric retention, hypoglycemia, and weight loss of less than 15 g/d of the premature infants in the FI group. ③ The digestive function after treatment in terms of daily increased breast milk volume, daily defecation frequency, and meconium emptying time was compared between group A and group B. ④ The observation indexes of the feeding intolerance including vomiting, abdominal distension, gastric retention, and hypoglycemia after treatment were compared between group A and group B, and the number of premature infants with those symptoms was recorded and calculated. ⑤ The treatment indexes including average length of hospital stay, sleeping time, and average increased weight were compared between group A and group B.

### 2.6. Statistical Treatment

We chose SPSS20.0 as the selected data processing software for this study, and GraphPad Prism 7 (GraphPad Software, San Diego, USA) was used to draw the pictures of the data. Measurement data were tested by *t*-test, while enumeration data were tested by *X*^2^ test. The differences had statistical significance when *P* < 0.05.

## 3. Results

### 3.1. Comparison of the General Information of the Premature Infants between the FI Group and the Control Group

The birthweight and gestational age of the premature infants in the FI group were significantly lower than those in the control group (*P* < 0.001), whereas there were no significant differences in other general information between the two groups (*P* > 0.05), as shown in Table 2.

### 3.2. Clinical Symptoms of the Premature Infants in the FI Group

In the FI group, the abdominal distension rate of the premature infants with the gestational age of less than 30 weeks was significantly higher than that of premature infants with other gestational ages (*P* < 0.05), the vomiting rate of the premature infants with the birthweight of more than 2500 g was significantly higher than that of premature infants with other birthweight (*P* < 0.05), and the incidence of abdominal distension and gastric retention of the premature infants with the breastfeeding initiation time of more than or equal to 72 h was significantly higher than that of the premature infants with the breastfeeding initiation time of less than 72 h (*P* < 0.05), as shown in Table 3.

### 3.3. Comparison of the Digestive Function of the Premature Infants between Group A and Group B after Treatment

The digestive function of the premature infants in group A after treatment was significantly better than that in group B (*P* < 0.05), with statistically significant differences, as shown in Table 4.

### 3.4. Comparison of the Observation Indexes of Intolerance between Group A and Group B after Treatment

The incidence of intolerance after treatment in group A was significantly lower than that in group B (*P* < 0.05), with statistically significant differences, as shown in Figure 1.

Note: the abscissa represented vomiting, abdominal distension, gastric retention, and hypoglycemia. In group A, there were 2 cases of vomiting, accounting for 6.7%, 3 cases of abdominal distension, accounting for 10.0%, 4 cases of gastric retention, accounting for 13.3%, and 1 case of hypoglycemia, accounting for 3.3%, with 10 cases and making up 33.3% in total, while in the group B, there were 5 cases of vomiting, accounting for 16.7%, 6 cases of abdominal distension, accounting for 20.0%, 6 cases of gastric retention, accounting for 20.0%, and 5 cases of hypoglycemia, accounting for 16.7%, with 22 cases and making up 73.3% in total.

### 3.5. Comparison of the Other Treatment Indexes between Group A and Group B

The daily gained weight of the premature infants in group A was (20.1 ± 1.2) g, which was significantly higher than that in group B (16.5 ± 1.5) g (*P* < 0.001); the premature infants in group A had shorter length of hospital stay and longer sleeping time as well as better treatment indexes than those in group B (*P* < 0.001), with statistically significant differences, as shown in Figure 2 for details.

Note: the abscissa represented average length of hospital stay and sleeping time. The average length of hospital stay and sleeping time of the premature infants in group A were (21.2 ± 2.1) d and (19.8 ± 1.2) d, respectively, while those in group B were (25.6 ± 2.0) d and (16.6 ± 1.5) d, respectively.^*∗*^ indicates *P* < 0.001.

## 4. Discussion

Our study results showed that in the FI group, the abdominal distension rate of the premature infants with the gestational age of less than 30 weeks was significantly higher than that of premature infants with other gestational ages (*P* < 0.05), the vomiting rate of the premature infants with the birthweight of more than 2500 g was significantly higher than that of premature infants with other birthweight (*P* < 0.05), and the incidence of abdominal distension and gastric retention of the premature infants with the breastfeeding initiation time of more than or equal to 72 h was significantly higher than that of the premature infants with the breastfeeding initiation time of less than 72 h (*P* < 0.05), all of these indicating that vomiting, abdominal distension, and gastric retention are the main clinical features of FI [16–19]. Foreign scholar, Hannah B, through analyzing the clinical symptoms of FI premature infants with different gestational ages and weights, has concluded that the premature infants with FI mostly present with abdominal distension and vomiting, and the abdominal distension rate of the premature infants with the gestational age of less than 30 weeks is 50.2%, suggesting that lower gestational age leads to higher abdominal distension rate [20], which is in line with our study results.

Traditional Chinese medicine holds that acupoint Zusanli dominates the basic function of internal organs, demonstrating that it is the preferred acupoint for the treatment of abdominal distension and the acupoint massage implemented on it has positive effect on promoting stomach intestine motility. Additionally, acupoint massage has the advantages of less irritation and more acceptability, thus it is a more desirable treatment modality [21–23]. In this study, the digestive function of the premature infants in group A after treatment was significantly better than that in group B (*P* < 0.05), and the average daily gained weight of the premature infants in group A was significantly higher than that in group B (*P* < 0.001). Group A had shorter length of hospital stay and longer sleep time than group B (*P* < 0.001), showing more obvious therapeutic effect in group A. Besides, the incidence of intolerance after treatment in group A was significantly lower than that in group B (*P* < 0.05), proving that combination therapy with acupoint massage on Zusanli can effectively relieve clinical symptoms such as abdominal distension and vomiting of the premature infants.

## 5. Conclusion

In conclusion, the clinical symptoms of premature infants with FI mainly include abdominal distension, vomiting, and gastric retention, and the incidence of each symptom varies in different infants, so the treatment should be carried out according to infants' own specific conditions. In addition, the application of acupoint massage on Zusanli combined with routine treatment can positively enhance gastrointestinal motility, improve digestive function, and relieve the clinical symptoms of premature infants, which is worthy of application and promotion in clinical practice.

## Figures and Tables

**Figure 1:** Comparison of the observation indexes of intolerance between group A and group B after treatment.

**Figure 2:** Comparison of the other treatment indexes between group A and group B.

**Table 1:** Comparison of the general information of the premature infants between group A and group B.

Group	Group A (*n* = 30)	Group B (*n* = 30)	**x** ^2^/**t**	*P* value
Gender			0.250	0.617
** **Male	15	17		
** **Female	15	13		
Gestational age	30.2 ± 2.1	30.5 ± 1.9	0.580	0.564
Birthweight	1258.1 ± 269.2	1258.5 ± 270.2	0.006	0.995
Apgar score	9.3 ± 0.2	9.3 ± 0.3	0.000	1.000
Anoxia after birth	No	No	——	——
Placenta	Normal	Normal	——	——
Delivery mode			0.074	0.785
** **Natural labor	14	13		
** **Cesarean delivery	16	17		
Perinatal infection	No	No	——	——

**Table 2:** Comparison of the general information of the premature infants between the FI group and the control group.

Group	FI group (*n* = 60)	Control group (*n* = 60)	**x** ^2^/**t**	*P* value
Gender			0.032	0.859
** **Male/female	32/28	31/29		
Gestational age (weeks)	30.4 ± 2.0	32.3 ± 1.8	5.470	≤0.001
Birthweight (g)	1258.1 ± 273.2	1486.5 ± 328.4	4.142	≤0.001
Maternal age (years old)	30.5 ± 1.5	30.6 ± 1.8	0.331	0.742
Delivery mode			0.036	0.849
** **Natural labor	27	28		
** **Cesarean delivery	33	32		
Complications during pregnancy			0.018	0.894
** **Yes	57	56		
** **No	3	4		

**Table 3:** Clinical symptoms of the premature infants in the FI group (n (%)).

Group	Types	Cases	Vomiting	Abdominal distension	Gastric retention	Hypoglycemia	Weight loss of more than 15 g/d
Gestational age (weeks)	＜30	21	4 (19.0)	11 (52.4)	10 (47.6)	5 (23.8)	4 (19.0)
	30–35	19	4 (21.1)	4 (21.1)	5 (26.3)	2 (10.5)	2 (10.5)
	36–37	20	9 (45.0)	4 (20.0)	7 (35.0)	2 (10.0)	2 (10.0)
Weight (g)	＜1500	25	8 (32.0)	12 (48.0)	6 (24.0)	3 (12.0)	3 (12.0)
	1500–2500	30	8 (26.7)	9 (30.0)	9 (30.0)	5 (16.7)	6 (20.0)
	＞2500	5	4 (80.0)	1 (20.0)	1 (20.0)	0 (0.0)	1 (20.0)
Breastfeeding initiation time (h)	≥72	32	10 (31.3)	15 (46.9)	15 (46.9)	3 (9.4)	2 (6.3)
	＜72	28	3 (10.7)	4 (14.3)	5 (17.9)	2 (7.1)	2 (7.1)

**Table 4:** Comparison of the digestive function of the premature infants between group A and group B after treatment ($\bar{x}$ ± *s*).

Group	*n*	Daily increased breast milk volume (ml)	Daily defecation frequency (times)	Meconium emptying time (d)
Group A	30	13.5 ± 3.2	3.8 ± 2.0	3.3 ± 0.2
Group B	30	11.0 ± 2.7	2.7 ± 0.5	4.1 ± 0.5
*t*		3.270	2.923	8.137
*P* value		0.002	0.005	<0.001

## Data Availability

The datasets used and/or analyzed during the current study are available from the corresponding author on reasonable request.
